# A systematic summary of survival and death signalling during the life of hair follicle stem cells

**DOI:** 10.1186/s13287-021-02527-y

**Published:** 2021-08-11

**Authors:** Xi-Min Hu, Zhi-Xin Li, Dan-Yi Zhang, Yi-Chao Yang, Shen-ao Fu, Zai-Qiu Zhang, Rong-Hua Yang, Kun Xiong

**Affiliations:** 1 Department of Anatomy and Neurobiology, School of Basic Medical Sciences, Central South University, Morphological Sciences Building, 172 Tongzi Po Road, Changsha, 410013 China; 2 Department of Dermatology, Xiangya Hospital, Central South University, Changsha, 410013 China; 3 Department of Burn Surgery, The First People’s Hospital of Foshan, #81, Lingnan North Road, Foshan, 528000 China; 4 Hunan Key Laboratory of Ophthalmology, Changsha, 410008 China

**Keywords:** Hair follicle stem cells (HFSCs), Signalling, Wnt, Shh, Notch, BMP, Apoptosis

## Abstract

Hair follicle stem cells (HFSCs) are among the most widely available resources and most frequently approved model systems used for studying adult stem cells. HFSCs are particularly useful because of their self-renewal and differentiation properties. Additionally, the cyclic growth of hair follicles is driven by HFSCs. There are high expectations for the use of HFSCs as favourable systems for studying the molecular mechanisms that contribute to HFSC identification and can be applied to hair loss therapy, such as the activation or regeneration of hair follicles, and to the generation of hair using a tissue-engineering strategy. A variety of molecules are involved in the networks that critically regulate the fate of HFSCs, such as factors in hair follicle growth and development (in the Wnt pathway, Sonic hedgehog pathway, Notch pathway, and BMP pathway), and that suppress apoptotic cues (the apoptosis pathway). Here, we review the life cycle, biomarkers and functions of HFSCs, concluding with a summary of the signalling pathways involved in HFSC fate for promoting better understanding of the pathophysiological changes in the HFSC niche. Importantly, we highlight the potential mechanisms underlying the therapeutic targets involved in pathways associated with the treatment of hair loss and other disorders of skin and hair, including alopecia, skin cancer, skin inflammation, and skin wound healing.

## Introduction

Hair contributes to a healthy life of human beings through their sensory effects, thermoregulation, physical protection, and social interaction impacts. In this regard, disorders of skin and hair, such as alopecia, anagen effluvium, telogen effluvium, hirsutism, hypertrichosis, and miniaturization, negative affect health [1]. Alopecia is a serious problem affecting 60–70% of the adult population worldwide, up to 70% of men and 40% of women, costing more than 3.5 billion every year in the U.S.A. [2, 3]. The regeneration of hair shafts produced by hair follicles (HFs) relies on the activation of a major reservoir of hair follicle stem cells (HFSCs), which is therefore utilized in stem cell-based therapy for treating alopecia.

The HF, a complex mini-organ of the skin, provides the stem cell (SC) microenvironment “niche”, functioning as a crucial regulator of cell fate by controlling the consecutive cycles of hair growth rest (the telogen phase), active hair growth (the anagen phase), and apoptotic-mediated hair growth regression (the catagen phase). This process depends on an elaborate network formed through multiple pathways, such as the Wnt/β-catenin pathway, Sonic hedgehog (Shh) pathway, Notch pathway, BMP (bone morphogenetic proteins) pathway and apoptotic pathway. Among these pathways, the Wnt/β-catenin signalling pathway plays a diverse role in initiating HFSCs for hair growth during hair regeneration [4]. Upregulation of Wnt10b or activation of Akt and Wnt/β-catenin can induce HFSCs to enter anagen from the telogen phase, resulting in accelerated hair regeneration [5, 6]. In addition, the proliferation of quiescent SCs can be induced by Shh pathway activation, and hair morphogenesis is closely related to Shh signalling [7]. Moreover, HFSC progeny secrete Shh, leading to the initiation of HF regeneration in adults [8]. The Notch pathway is a major mechanistic pathway in the fate determination of HFSCs, and the Maria group and Niwa group showed that Notch signalling promoted HFSC activation in a regulatory T cell (Treg)-mediated manner [9, 10]. Furthermore, BMP signalling is regarded as a suppressant of HFSC activity, whereas TGF-β2 signalling can antagonize BMP signalling to promote HF regeneration [11]. Apoptotic signalling is also vital for the pathological (*e.g*., following radiation-induced damage) and physiological (*e.g*., catagen phase) processes in which molecules known as caspase or Bcl-2 are activated [12]. Through a unique molecular mechanism, each of these proteins exerts special functions, while complex connections are established between them. For example, BMP signalling is not activated at the same time as the Wnt/β-catenin signalling pathway, but the Wnt pathway can be inhibited by BMP expression, and sustained Shh expression relies on BMP inhibition [13, 14].

HFSCs have been shown to differentiate into nerve cells, glial cells, keratinocytes, smooth muscle cells, cardiac muscle cells, and melanocytes, which suggests tremendous potential for HFSCs as targets in the treatment of various diseases. Genetic profiling of HFSCs has revealed several known and previously unknown molecules and signalling pathways, including those involved not only in survival but also in death mechanisms, which are important for maintaining the SC phenotype. Ultimately, these findings indicate a number of potential targets for the treatment of hair loss and other skin and hair disorders.

## A brief introduction to HFSCs

### HFSC status in the hair cycle and niche microenvironment

An HF is known as a complex mini-organ embedded in the skin that is formed by the papilla, matrix, root sheath and bulge. And the tissue homeostasis in HFs and their damage repair rely on a variety of stem cells within the HFs, including HFSCs mostly located in the hair follicle bulge, keratinocyte progenitor cells from the hair follicle bulge area, melanocyte progenitor cells, nestin-expressing stem cells, skin-derived precursors (SKPs) located in the DP, and also stem cells in eccrine gland and sebaceous gland [15–20]. HFSCs constitute the major portion of SCs in HFs, which are derived from the neuroectoderm and exhibit the potential to differentiate into multiple cell types [21]. Due to the discovery of HFSCs, we have made a deeper insight into the growth, development and regulation of HFs [16, 22, 23]. And the term ‘HFSCs’ was first coined in 1990s, which is first identified in the bulge epithelium as label-retaining cells (LRCs) [16].

During HF cycling (the telogen, anagen, and catagen phases) and/or injury repair, HFSCs may remain quiescent continuously or acquire a different status, engaging the mechanism(s) to respond to their own niche microenvironment. In the telogen phase, HFSCs are located in the bulge and maintain quiescence because of various inhibiting factors. The dermal papilla (DP) is located immediately below the bulge, and it can secrete factors to regulate the state of HFSCs. Once a critical concentration of SC activators has been reached, a subset of HFSCs is activated, and the anagen phase is initiated [24]. Interestingly, only a small number of HFSCs near the DP undergo asymmetric division and become transient amplifying cells (TACs). The remaining HFSCs remain in the bulge and maintain quiescence. In the anagen phase, TACs differentiate into the matrix and sheath of a hair shaft, forming the lower part of an HF [1]. Then, the bulge and DP gradually move away. During the catagen phase, the lower two-thirds of the HF rapidly regress. The lower HF is reduced to an epithelial strand, bringing the dermal papilla into close proximity of the bulge [25]. The signalling molecules that regulate HFSCs are mainly derived from the DP.

With the regulation of the HFSC life cycle, a complex and vital element may point to the niche as well as to the other microenvironments (including dermal papilla, adipose tissue, lymphatic vessels, nerves and immune cells, etc.) [26]. For example, a vast amount of lipids are stored in mature adipocytes and supply energy for SC proliferation and rapid hair production/elongation [27]. A detailed review of the molecular pathways involved in HFSCs is presented herein.

### Specific markers of HFSCs and the HF structure

To identify and separate HFSCs from other HF cells, knowing their location and the specific markers is necessary [28]. The longitudinal surface of an HF can be divided into three parts from the epidermis to deep layers: the infundibulum (from the surface of the skin to the duct of the sebaceous gland), the isthmus (from the duct of the sebaceous gland to the attachment of the arrector pili muscle, APM) and the hair bulb (below the attached APM). It can also be divided in the horizontal direction; that is, the HF consists of an inner root sheath (IRS), which includes Henle’s layer, Huxley’s layer, the cuticle layer, the companion layer, and the outer root sheath (ORS), which contains keratinocytes, melanocyte stem cells, etc. The prominent bulge between the APM attached to the ORS and the sebaceous gland duct is the reservoir of human HFSCs (hHFSCs) [1, 29, 30]. We provide a figure of the HF structure and the specific markers of HFSCs (Fig. 1).

**Fig. 1:** Structure of the hair follicle and specific markers in HFSCs

With further research on hHFSCs in recent years, the accurate identification of hHFSCs has become an important problem to be solved. Due to the complexity of the HF structure and cell composition, it is generally believed that a combination of multiple markers should be used to identify HFSCs in the bulge.

CK15 was one of the first identified hHFSC markers and is expressed in all stages of human bulge cells [31–33]. It has been widely used in identifying hHFSCs and is considered to be one of the best markers of hHFSCs [30, 34, 35]. However, CK15 was also found to be continuously expressed in the basal epidermal layer, sweat glands and oral epithelial cells, which raised concerns about the reliability of using CK15 as a marker of hHFSCs [36, 37]. First, integrin β-1 was found to be coexpressed with CK15 in hHFSCs of bulge [31, 32, 38]. However, later studies showed that integrin β-1 is not expressed more intensively in the bulge than in the adjacent ORS [34, 39]. Therefore, identification of CK15 should be used with the identification of other markers to identify hHFSCs.

CK19 is another positive marker that has been widely used for the identification of hHFSCs [31, 34, 38] and is expressed in the anagen and telogen phases of the HF cycle [40]. However, during differentiation, CK19 expression decreases later than CK15 expression, and CK19 is also expressed in ORS cells below the bulge area in an HF [31, 41]. An interesting hypothesis suggests that CK19-positive cells in the bulge region are derived from CK15-positive cells. Only CK15-positive cells are found above the area of the HF in which both CK15-positive and CK19-positive cells are located, and conversely, only CK19-positive cells are located below the area where both CK15-positive and CK19-positive cells are found [42]. Hence, CK15 may be a better marker for identifying hHFSCs.

CD200 is another positive marker commonly used for the identification of hHFSCs [30, 39, 43]. Ohyama et al. successfully obtained HF bulge region stem cells from human HF suspensions using CD200 as a positive marker. In addition, pleckstrin homology-like domain family A member 1 (PHLDA1), also called T cell death-associated gene 51 (TDAG51), can prevent apoptosis. A gene microarray analysis showed that *PHLDA1* was preferentially located in the bulge cells of the ORS at both the mRNA and protein levels [43]. According to an immunohistochemical analysis, PHLDA1 was also found in the follicle bulge [44]. Nevertheless, *PHLDA1* is not specifically expressed in hHFSCs; it can also be expressed in sweat glands and epidermal melanocytes [45]. Furthermore, NFATC1 was found to be expressed in SCs in HF bulges [46]. EpCAM/BER-EP4 is considered to be a useful marker of the telogen optional hair germ [47].

CD34 is a specific positive marker of mouse follicle stem cells [48, 49]. However, in hHFSCs, CD34-positive cells are expressed below the bulge region and only expressed during the anagen phase. The expression of CD34 in cells of the bulge region in human HFs is low or absent [43, 50]. CD24-positive cells are not characteristic of HFSCs and are therefore considered to be a negative marker [43]. Lgr6 have been utilized to mark the most primitive epidermal stem cell, and Lgr6 connected with its close relative- Lgr5 has also used as a biomarker of HFSCs [51, 52]. Also, nestin, an intermediate filament protein, could serve as a marker of HFSCs, and also neural stem cell [53]. Cells, located in the HF pluripotent stem cell (hfPS) area (hfPSA), could be labelled with the nestin positive and keratin 15 (K15)^−^ negative [53]. Other markers of hHFSCs have been identified, including CD71 [43], CD146 [43], Connexin 43 [34], Sca-1 [54], Bcrp1 [54], and P75NTR [54, 55]. In order to improve the accuracy of detection of HFSCs, recent studies have made use of a combination of a body of markers to identify HFSCs.

Horizontally (in the horizontal direction), the HF consists of the inner root sheath (IRS) the companion layer, and the outer root sheath (ORS). The structure of the hair follicle is formed by some of the contents: dermal papilla (DP) as dermal part of the hair follicle; inner root sheath (IRS) as the inner channel of the hair shaft which locates various of stem cells such as HFSC; hair shaft: emerging as a hair from the skin surface; outer root sheath (ORS): the external layer of the HF. A prominent bulge between the APM of the ORS and the duct of the sebaceous gland is considered to be the reservoir of human HFSCs (hHFSCs). Here, the location and multiple markers of HFSCs are shown in the figure.

### HFSC functions and applications

For an in-depth exploration of HFSCs, understanding the functions of HFSCs will contribute to the useful parameters for both further study and clinical applications. On the one hand, HFSCs have the ability to self-renew and differentiate into ectodermal and mesodermal cell lineages during injury repair, forming abundant and enriched pools of cells involved in repair. HFSCs contribute to tissue homeostasis in HFs [56], and HFSCs can also promote cutaneous wound healing via different pathways, such as through the high expression of SDF-1α and CXCR4 [57]. In addition, they have the potential to differentiate into many kinds of cells, such as neurons, Schwann cells, melanocytes, keratinocytes, adipocytes, smooth muscle cells, and bone cells [15, 18, 58, 59]. Considering this ability, some studies have shown that injection of HFSC exerted a protective influence on middle cerebral artery ischaemia/reperfusion due to the regeneration of neurons and the reduction in infarct volume in rat models [60]. The large capacity for self-renewal and differentiation into most mesodermal and ectodermal cell derivatives makes HFSCs prominent among all SCs. Along with the rapid development of SC technologies, we believe that activating HFSCs may hold promise for the therapy of many kinds of diseases, such as cardiovascular diseases and motor system diseases.

On the other hand, HFSCs can influence multiple other cells or tissues. For example, HFSCs enhanced tissue tensile strength as vascular density increases in an HFSC-treated animal model of burn wounds [61]. In addition, some factors secreted from HFSCs play significant roles in modulating surrounding niche cells. For instance, signals from HFSCs can regulate the surrounding skin vasculature. HFSC-derived Angptl7 transcription is involved in lymphatic dynamics, and HFSCs can remodel the vasculature around the HF by changing Runx1 levels [62, 63]. In summary, HFSCs contribute not only to renewal and reestablishment of HFs but also to the regulation of niche homeostasis.

## Signals and signaling pathways in HFSCs

The fate and functions of SCs related to tissue renewal, regeneration, and development are rigorously controlled by the local microenvironment (also known as the “niche”, which is formed by various biomolecules such as cytokines, growth factors and others) via a complex signalling network [4, 64, 65]. Damage and protective factors participate as initiators in these signalling pathways during the development and pathology of HFSCs. Damage inducers include mechanical force, ultraviolet (UV)-induced stress, drug-induced stress, hormonal disorders or dihydrotestosterone (DHT) damage (inducing androgenic alopecia), and psychological stress [4, 48, 66, 67]. Protective factors include platelet-rich plasma (PRP), an adequate supply of oxygen and blood, etc. [68]. The regulation of survival and death signalling pathways plays a driving role in the quiescence, activation, differentiation and metabolism of HFSCs, which is fundamental for skin homeostasis, hair repair, and hair growth. We review the major signalling pathways that are activated during the life of HFSCs, including during survival and death.

### Molecular mechanisms affecting the survival of HFSCs

#### The Wnt/β-catenin pathway

Wnt is in a family of extracellular developmental signalling proteins controlling a myriad of different cellular fates [69]. For example, the activation of Wnt/β-catenin can promote the continuation of the process of renewal of various tissues by fuelling SC activity [14]. The canonical Wnt/β-catenin pathway is mainly related to a class of Wnt hydrophobic proteins tethered to their cognate receptors on the cell membrane, driving a series of transcriptional programmes (Fig. 2). The processes of Wnt pathways are shown and discussed in further detail below.

**Fig. 2:** Molecular mechanisms and functions of the Wnt/β-catenin signalling pathway in HFSCs. **a** In the absence of a Wnt signal for the binding of Wnt inhibitors (*e.g*., sFRP1, Dkk3, or Wif), a multiprotein complex is formed with APC, Axin, and GSK3, which can target and phosphorylate β-catenin, leading to excessive cytoplasmic β-catenin degradation. **b** Once Wnt binds to Frizzled and lipoprotein receptor-related protein (Lrp5/6 receptors), the activated receptor complex induces recruitment of certain key components, such as Dvl, which results in the destruction complex disassembling, to prevent β-catenin degradation. Accumulated and stabilized β-catenin is translocated to the nucleus, where it can bind transcription factors (*e.g*., LEF/TCF family) to promote the expression of target genes, such as *Axin2*, *LEF1* and *Lgr5*. **c** Wnt signalling shows a close association with HFSCs in quiescence, activation, and differentiation and even in Wnt-induced tumorigenesis. The T-shaped lines indicate inhibitory interactions involved in this pathway, and the solid arrows indicate activating interactions

As early as the 1990s, transgenic mouse studies revealed the diverse roles of Wnt signalling in the specific development of HFs; specifically, de novo follicles were shown to express stabilized β-catenin in mice, and few follicles were found in mice lacking Lef1 or β-catenin [70, 71]. With the development of in-depth mechanistic studies, a detailed molecular pathway was shown more clearly both in terms of the activation and inhibition of Wnt signalling. In the absence of a Wnt signal, a multiprotein complex formed by APC, Axin, and GSK3 can target and phosphorylate β-catenin, leading to excessive cytoplasmic β-catenin degradation. It has been reported that upregulation of DKK1, IWP2, or sFRP1 (a specific negative regulator of Wnt signalling) can inhibit accelerated HFSC proliferation and differentiation into follicular components [6, 72, 73]. Normally, the bulge is observed in a Wnt-inhibited environment, as microarray data have shown that the genes encoding putative Wnt inhibitors (*e.g*., *sFRP1, Dkk3,* and *Wif*) are upregulated and that the genes encoding Wnt promotors (*e.g*., *Wnt3* and *Wnt3a*) are downregulated [23]. However, this quiescence needs to be disrupted at certain times through bulge SCs expressing a number of surface Wnt signal receptors (*e.g*., *frizzled 2/3/7*) to enable a combination of Wnt signals [23].

Once Wnt binds to Frizzled and lipoprotein receptor-related protein (Lrp5/6 receptors), the activated receptor complex induces recruitment of certain key components, such as Dvl (Disheveled), which results in the destruction complex disassembling, preventing β-catenin degradation. Wnt10b, a canonical Wnt ligands, has been shown to be upregulated in the secondary hair germ region, where the expression of β-catenin is overregulated upon anagen phase onset, highly expressed in the middle anagen phase, and expressed at low levels in the catagen and telogen phases, whereas the absence of β-catenin signalling in the skin leads o inhibited hair regeneration and permanent hair loss [70, 74]. Wnt10b functions as a major activator, and Wnt10b is an activator that regulates HFSC expression during the telogen-anagen phase transition [75].

The mechanism that stabilizes β-catenin during HFSC development leads to a change in the telogen-to-anagen transition of the hair cycle. Accumulated and stabilized β-catenin is translocated to the nucleus, where it can bind transcription factors (*e.g*., LEF/TCF family) to promote the expression of target genes, such as *Axin2*, *LEF1* and *Lgr5,* resulting in the promotion of TAC conversion, and is replaced in activated cells during de novo follicle generation (Fig. 2) [76, 77]. Some groups have reported that activation of hair regeneration occurs precociously upon the upregulation of stabilized β-catenin expression in the telogen phase [77]. Additionally, a microarray assay showed transgene expression changes (*e.g*., in *Sox4*, *biglycan*, and *cyclin D2* (*Ccnd2*)) in telogen- or anagen-phase SCs isolated from β-catenin-mutant or wild-type follicles, which may promote hair cycle progression [77]. This signalling seems to emanate from the DP in close proximity to the bulge. Consistent with this notion, some studies have found that exosomes derived from DP cells can promote the anagen phase of HFs [78].

Overall, the Wnt/β-catenin pathway has been considered a central signalling pathway leading to the transition of HFs from the telogen to anagen phase, which is closely related to the physiology and pathology of other skin components, such as HF morphogenesis, hair shaft differentiation, and pathological changes (*e.g*., pilomatricoma tumour induction) [79–81].

#### The Sonic hedgehog (Shh) pathway

The Shh pathway plays a driving role in regulating developmental patterning and proliferation in multiple tissues, including HF tissue [82, 83]. This connection with HFs can be traced to two direct functions of Shh: 1) improving quiescent SC proliferation and 2) regulating the dermal factors that induce TAC expansion [7]. Quiescent SCs begin to express Shh, while primed SCs generate TACs, and it has been found that the TAC pool is reduced in the absence of Shh signalling [7].

In addition to the Wnt pathway, the development of HFSCs is also linked to Shh signalling, as shown in Fig. 3. In the Shh signalling pathway, Shh induces the release of inhibition of Smoothened (Smo, a G protein-coupled receptor (GPCR)-like protein). Subsequently, Smo can translocate into the membrane and initiate the activation and translocation of Gli into the nucleus, allowing the transcription of target genes (*e.g*., *Ptch* and *Gli1*) forming a feedback loop in this pathway [84–86]. When the ligand Shh does not bind to its receptor Patched (PTCH), this cascade reaction is aborted because Gli is sequestered in the cytoplasm via its interaction with suppressor of fused homologue (Sufu, one of the crucial inhibitors during Shh signalling) [87]. In other words, PTCH is an inhibitor leading to repression of Shh pathway activation, whereas basal cell carcinoma (BCC), featuring frequent loss of PTCH expression, can cause constitutive activation of the Shh pathway [88, 89]. Shelby et al*.* found that multiple HFSC populations readily develop into BCC-like tumours in *Ptch1*-deleted mice [88], and Kasper et al. reported that more than 90% of human BCCs are thought to be caused by loss of PTCH1 [90]. Additionally, overexpression of Shh, Smo, or Gli1/2 has been identified during BCC development [91, 92]. Interestingly, HFSCs can also emerge as regulators through the Shh signalling pathway during the development of tissue, which in turn controls HFSC regeneration. HFSCs secrete Shh to direct the formation of the APM-sympathetic nerve niche, forming form a dual-component niche for HFSCs [8].

**Fig. 3:** The Shh signalling pathway in HFSCs. **a** In the absence of Shh, the complex consisting of Gli and Sufu cannot form, preventing the transcription of the target genes. **b** In the Shh pathway, Shh induces the release of Smo inhibition. Then, Smo can translocate into the membrane and initiate the activation and translocation of Gli into the nucleus, allowing the transcription of target genes (*e.g*., *Ptch* and *Gli1*), creating a feedback loop in this pathway. When the Shh ligand does not bind to its receptor, PTCH, this cascade is aborted, and Gli is sequestered in the cytoplasm via the interaction with suppressor of fused homologue (Sufu, one of the crucial inhibitors of Shh signalling). The T-shaped lines indicate inhibitory interactions involved in this pathway, and the solid arrows indicate activating interactions

Shh signalling enriches the pathways activated in HFSC development. However, it remains unclear how signalling and cell diversity function during the hair cycle. Both signals form a bud (a hair germ), as it still occurs in the absence of Shh signalling [93].

#### The Notch pathway

During the maintenance of self-renewal in multiple tissues, Notch signalling is closely related to the promotion or suppression of cell proliferation, failure of differentiation programmes, or cell fates. Additionally, many studies have reported a connection between Notch signalling and hair health and hair-related diseases [14]. For example, upregulated and active Notch1 has been found in basal and suprabasal cells in sebaceous glands during the early stage of epidermal stratification; a reduction in the number of HFs occurs in the absence of Notch1 signalling; and Notch1-3 have been identified in differentiating HF cells [94–96]. Aiming to explain how Notch signalling acts in the hair cycle, further research has focused on Notch signalling in the bulge SC niche to influence SC maintenance and activation.

Similar to the signalling mentioned above, the Notch pathway also contributes to a certain protein translocating to the nucleus and activating downstream target genes to affect cellular metabolism and growth (shown in Fig. 4) [97]. First, a fully functional Notch receptor binds to a ligand (Dll1-4 or Jag1-2) presented by a neighbouring cell. Once induced, the conformational change of the receptor exposes the recognition site to cleavage by ADAM (a disintegrin and metalloprotease) and γ-secretase, which leads to the release of the active Notch intracellular domain (NICD). A high level of Notch ligand family member-Jagged 1 (Jag1), which induces the activation, proliferation and differentiation of HFSCs in newly generated HFs in the hair cycle, was identified in Tregs [9, 10]. Then, NICD is translocated to the nucleus, leading to the formation of a tri-protein complex, consisting of the DNA-binding CSL complex (consisting of CBF1/RBPjκ/Su(H)/lag-1)/additional coactivators (Co-A)/mastermind (MAM), which induces the transcription of target genes. Conditional disruption the mouse *RBP-J* gene can cause hair loss and epidermal cyst formation via the aberrant differentiation of RBP-deficient HFSCs [98]. Without the activation of Notch signalling, the NICD does not enter the nucleus, and CSL might connect with ubiquitous corepressor (Co-R) proteins and histone deacetylases (HDACs) to repress target gene transcription. Interestingly, Notch associated with cofactor RBP-J can also function in HFSCs to suppress downstream genes such as retinoid metabolic process genes, which reveals a previously unknown role of Notch signalling in regulating metabolites in HFSCs [99].

**Fig. 4:** The Notch signalling pathway in HFSCs. **a** Without the activation of Notch, the NICD does not enter the nucleus, and CSL might connect with ubiquitous corepressors (Co-R) and histone deacetylases (HDACs) to repress target gene transcription. **b** In the Notch pathway, a fully functional Notch receptor binds to a ligand (Dll1-4 or Jag1-2) presented by a neighbouring cell, resulting in a conformational change of the receptor that expose the recognition site for cleavage by ADAM and γ-secretase, leading to the release of the active Notch intracellular domain (NICD). Subsequently, NICD is translocated to the nucleus, leading to the formation of a complex, the DNA-binding protein CSL (CBF1/RBPjκ/Su(H)/lag-1)/additional coactivators (Co-A)/mastermind (MAM), which induces the transcription of target genes. **c** Notch signalling plays a vital role in the activation, proliferation, deafferentation of HFSCs and metabolite generation. The T-shaped lines indicate inhibitory interactions involved in this pathway, and the solid arrows indicate activating interactions

A number of studies have shown Notch signalling in HF morphogenesis and gradually revealing this Notch signalling pathway in HFSCs, attracting the interest of scientists seeking to explain the mechanism of the Notch signalling axis, and further research is needed to determine the complex downstream genes regulated by Notch signalling in HFSCs, the association of Notch with other signalling molecules in co-networks in HFSCs that influence the hair cycle, and to determine whether these proteins and/or genes are stable and effective targets for clinical application.

#### Bone morphogenetic protein (BMP) pathway

HFSCs, particularly TAC formation in response to BMP signalling during a specific period of the hair cycle, exhibit self-regulated proliferation and differentiation [100]. BMPs, as a member of the TGF-β superfamily, exhibits biological activity after secretion and binding to a transmembrane heterodimeric receptor complex (formed by BMPR-I and BMPR-II) [83]. BMP signalling is a key mechanism that modulates or reinforces the quiescence of HFSCs upon self-renewal, maintains cell identity and is required for TAC generation [101, 102]. However, reduced or inhibited BMP signalling can also activate HFSCs; a loss of *Bmpr1a* in mice caused aberrant activation of quiescent HFSCs [101, 103, 104]. The expression of Noggin (a specific BMP antagonist) is upregulated upon mesenchymal condensation, while BMP is downregulated in the early stage of the hair cycle, which is required for HF activation and morphogenesis [13]. Recently, microRNAs (miRNAs, miRs) have been shown to be inhibitors of BMP signalling, and it has been reported that miR-29a/b1 can negatively regulate *Bmpr1a* by binding to the 3′-UTR of *Bmpr1a* [104].

The detailed mechanism of the BMP pathway is graphically presented in Fig. 5 and explains as follows: Upon initiation of the BMP pathway, a BMP dimer connects with a specific receptor. Then, the dimer phosphorylates and activates R-Smad (Smads 1/5/8) and subsequently associates with the co-Smad partner Smad 4 [101]. Finally, the complex formed by R-Smad/co-Smad is translocated into the nucleus, resulting in the transactivation of its target genes. However, the detailed mechanisms and biological functions of these downstream targets are still being discovered, and BMP signalling is likely to be involved in HFSCs in the HF cycle and HF morphogenesis. To gain insight, the Kandyba group utilized the keratin 15 (K15) promoter, driving inducible Cre recombinase to ablate *Bmpr1a* in telogen-phase HFSCs in the bulge and hair germ (HG). Then, this group found 16 upregulated RNAs (*e.g*., *Wnt7a/7b*/*16*) and 80 downregulated mRNAs (*e.g*., BMP6, FGF18 and Wnt inhibitor DKK3), which suggests a significant role for BMP in HFSCs closely related to the HF cycle [101, 105].

**Fig. 5:** The BMP signalling pathway in HFSCs. The BMP pathway is initiated by a BMP dimer connecting with a specific receptor. Then, the dimer phosphorylates and activates R-Smad (Smads 1/5/8), which subsequently associate with the co-Smad partner Smad 4. The T-shaped lines indicate inhibitory interactions involved in this pathway, and the solid arrows indicate activating interactions

In addition, Noggin/BMP signalling has also been found to play vital roles in lung alveolar stem cells and neural stem cells [106, 107]. Other inhibiting signalling, such as inhibition of the epidermal growth factor receptor (EGFR), contributes to the delicate balance between activation and quiescence during the development of HFSCs. Data have shown that in EGFR-knockout follicles, an elevated level of Wnt/6/7b/10a/10b and 16 transcripts and hyperactivation of β-catenin signalling [73].

#### The crosstalk between survival signalling pathways

Each signalling pathway discussed thus far has emerged as a regulator involved in the fate of HFSCs. Furthermore, a body of evidence suggests that more than one of these pathways is active in HFSCs, either at the same time or in different periods [93]. And a figure described crosstalk among the survival signalling pathways has shown in Fig. 6 Regarding the established links to both Wnt and Shh signalling, two interactive pathways have been described: (1) downstream glycogen synthase kinase-3β (GSK-3β) forms an complex inhibiting the Wnt and Shh morphogenetic pathways [108]; Notably, GSK3β is also an inhibitor of Notch signalling [109]. In contrast to other pathways, GSK3β contributes to Wnt signalling in an indirect way, as its phosphorylation at the N-terminal domain of β-catenin is mediated by the SC factor/ubiquitin/proteasome pathway, which is a key factor in Wnt signalling [110]. Once GSK3β is overexpressed, the pathways are inhibited, as is the differentiation of HFSCs; through one of the Shh positively regulated downstream genes, which can inhibit Wnt ligands and/or their receptors (namely, secreted frizzled-related protein-1 (sFRP-1)) or promote the Wnt process via Gli- and Fox- family, leading to either Wnt-Shh antagonistic or synergetic effects in the HFSCs [111]. Although both signals occur within the bud, the Shh pathway has been found to be genetically downstream of the Wnt pathway and is still activated in the absence of Shh; however, hair buds do not progress further [93, 112].

**Fig. 6:** The crosstalk among the survival signaling pathways. Each of the signals emerge as the regulators involved in the fate of HFSCs and these pathways (Notch, BMP, Wnt, Shh*, *etc*.*) emerge as a network in the life of HFSCs at the same time or in different period. Such as Dlx3, it is a homeobox transcription factor which could not only place downstream of Wnt through Lef targeting and causing a loss of BMP signaling. Moreover, Shh could up-regulate dermal noggin expression; which is a potent inhibitor of BMP signaling. The solid arrows indicate the targeting work from one of molecules involved in the signaling targeting to other signal pathways

Some molecular agents may establish the connections within this network in HFSCs or contribute to the development of hair. Dlx3 is a homeobox transcription factor that is not only activated downstream of Wnt through Lef targeting but is also the cause of lost BMP signalling. In the telogen phase bulge, HFSCs are inhibited to preclude reinitiation of the HF growth cycle upon the ablation of Dlx3 expression associated with Wnt signalling and a loss of BMP signalling [113]. The expression of *Shh* and *Sox*4 (a downstream target genes in the Wnt signalling pathway), characteristic of quiescent bulge cells and/or their early proliferating progeny, was upregulated after BMP pathway inhibition, controlling HFSC differentiation [70]. Lef1/β-catenin-mediated transcription in Wnt signalling is elevated in the absence of BMPR1A [114]. Moreover, dermal Shh can upregulate dermal noggin expression, which is a potent inhibitor of BMP signalling that helps to counteract BMP-mediated β-catenin inhibition [83].

Remarkably, an increasing number of signalling pathways related to HFSCs have been identified (shown in Table 1), and this co-network may involve these signalling pathways. For example, Notch signalling can suppress TGF-β and activate the Kit ligand to maintain an optimal matrix-proliferating environment for SCs [115, 116]. Moreover, mice lacking EGFR show overexpression of Wnts by upregulating the Wnt antagonist sFRP1, which coordinates the delicate balance between proliferation and differentiation during HFSC development [73]. Overall, the interactions are complex and involve multiple networks, not one crucial pathway, whose balance is vital to the fate and development of HFSCs.

**Table 1:** The survival signaling pathway in HFSCs

Signaling pathway	Axis	Key molecule	Regulation (up/down)	Target genes	Effects	Ref
Wnt	Wnt/β-catenin	Wnt	up	*Cyclin D1*	Initiating DNA synthesis and leading to the increase of viability of HFSCs	[117]
				*Myc*	Leading to the activation of HFSCs by increasing lactate production, and also increasing the viability of HFSCs	[117, 118]
				*Axin2*	Contributing to proliferation, migration of dermal papilla and promoting HFs growth	[119]
				*Lef1*	Activating target gene expression, promoting the activation, proliferation, and differentiation of HFSCs, increasing Shh level by leading to the downregulation of E-cadherin, and transmitting the early Wnt signals along with β-catenin	[6, 83, 120]
			down	*Dlx3*	Leading to enhanced proliferation and delayed regression, since it is essential in hair morphogenesis, differentiation and cycling programs, and also leading to the loss of BMP signaling	[83]
Shh	Msi2-Shh-Gli1	SHH	up	*Gli1*	Leading to HFSCs proliferation and differentiation, and inducing HFs neogenesis and hair placode/germ formation	[3, 121]
				*Ptch1*	Activating Gli1 transcription factors and leading to HFSCs proliferation and differentiation	[7]
				*Cyclin D1, Cyclin D2*	Inducing the activation of HFSCs and leading to the increase of viability of HFSCs	[7, 117]
				*Sox9*	Being required for SOX9( +) cell specification to HFSCs, leading to the production of Merkel cells in hair placode and maintaining the growth of HFs after morphogenesis	[122, 123]
Notch		NICD	up	*Hey1*	Leading to HFSCs proliferation	[99]
				*Hes1*	Replenish HFSCs in order to maintain the hair cycle homeostasis and leading to the activation of the secondary hair germ	[124]
				*Hes5*	Reducing HFSCs migration and clonogenicity	[125]
BMP		BMPR	up	*PTEN*	Inducing autophagy to facilitate HFSCs differentiation, inhibiting HFs hyperplasia and reducing the risk of tumorigenesis	[126, 127]
				*bHLH*	Being able to encode ID proteins as mediators of HFSCs quiescence	[128]
			down	*Wnt7b*	Leading to the disrupted HF cycling which manifests a shortening growth phase, premature catagen onset and shortening hair coat production with low-level expression of HFs differentiation markers	[129]
				*Lhx2*	Leading to the delay of HFSCs activation	[83]
TGF-β	TGF-β/smad	TGF-β	up	*Wnt*	Contributing to promotion of cells cycle for HFSCs	[117]
				*β-catenin*	Promoting the HFSCs proliferation and differentiation, and exerting long-term homeostasis of skin epithelia	[117, 120]
				*pSmad2*	Promoting the transition between telogen and anagen	[130]
				*Tmeff1*	Lowering the BMP threshold for HFSCs activation by mediating the inhibited effect of TGF-β2 on BMP signaling, and contributing in HFSCs activation during the telogen to anagen transition	[130]
EGFR	TGF-α/EGFR	EGFR	up	*TGM*	Leading to the differentiation of suprabasal-like KC and promoting cornified envelope formation	[131]
				*Flg*	Leading to the differentiation of HFSCs and contributing to the epidermal barrier function	[132]
			down	*Keratin 1*	Leading to the differentiation of suprabasal-like KC	[131]
				*Loricrin*	Leading to the differentiation of suprabasal-like KC	[131]
				*Wnt4*, *6*, *7b*, *10a*, *10b*	Being essential to restrain proliferation and support HFSCs numbers and their quiescence by influencing Wnt signal pathway	[133]
AKT	PI3K/AKT	AKT	up	*TGF-β2*	Leading to the activation of TGF-β mediated transcription in HFSCs and inducing HFSCs to proliferate during the quiescent period of the hair cycle	[130, 134]
				*IGFBP-3, 4, 24, and 25*	Exerting both growth-inhibitory and -potentiating effects for HFSCs, and IGFBP4 acting as an inhibitor in the canonical Wnt pathway by directly interacting with the Wnt receptor to prevent Wnt3a binding	[134]
			down	*IGFR1 and IGFR2*	Expressing a duality of HFSCs including both growth-inhibitory and -potentiating effects, and leading to delay in the anagen/catagen switch among HFs	[134, 135]
				*Fgf18*	Leading to HFSCs proliferation and hair regeneration	[6, 8]
				*Foxp1*	Leading to HFSCs proliferation and hair regeneration	[8]
Fox		Fox family protein	up	*Cdh1*	Weakening proliferative activity of Bu-HFSCs due to E-cadherin–mediated inter-SC adhesion	[136]
				*Lhx2*	Leading to HFSCs activation, maintaining their characters of regeneration and undifferentiation in HFs, and also promoting epidermal regeneration	[83, 137–139]
		LHX2	up	*Sox9*	Leading to HFSCs differentiation to promote epidermal regeneration in wound-healing process	[138]
				*Tcf4*	Leading to HFSCs differentiation to promote epidermal regeneration in wound-healing process	[138]
			down	*Lgr5*	Inhibiting the proliferation of HFSCs and disturbing the cycling of anagen HFs	[127, 138]

*Axin2* Axis inhibition protein 2, *bHLH* Basic helix-loop-helix, *BMP* Bone morphogenetic protein, *BMPR* Bone morphogenetic protein receptor, *Cdh* congenital diaphragmatic hernia; Distal-less homeobox, *EGFR* Epidermal Growth Factor Receptor, *Fgf* fibroblast growth factor, *Flg* filaggrin, *Fox* Forkhead box, *Foxp1* forkhead box protein 1, *Gli* Glioma-associated oncogene homolog, *Hes* Hairy enhancer of the split, *Hey* Hairy/enhancer-of-split related with YRPW motif, *IGFBP* Insulin-like growth factor-binding protein, *IGFR* insulin-like growth factor, *KC* keratinocytes, *Lef* Lymphoid enhancer-binding factor, *Lgr* leucine-rich repeat-containing G protein-coupled receptor, *Lhx* LIM homeobox, *NICD* Notch intracellular domain, *Ptch1* Patched-1, *PTEN* Phosphatase and tensin homolog, *SC* stem cell, *Shh* Sonic hedgehog, *Sox* SRY-related high-mobility-group box, *Tcf* T-cell factor, *TGF-α* Transforming growth factor-α, *TGF-β* Transforming growth factor-beta, *TGM* transglutaminase, *Tmeff1* Tomoregulin-1

### Molecular mechanisms during HFSC death

During the development of biological systems, tissue structures and organs are repaired and sculpted by the removal and addition of constituent cells via the alternative processes of controlled cell death (also known as regulated cell death, RCD, including apoptosis, autophagy, necroptosis, pyroptosis, and ferroptosis) and cell recruitment [140, 141]. In inferior HFs, RCD may be a central element of growth cycle progression and regression of each hair cycle [142]. Moreover, RCD occurs extensively in HFs during skin disorders in alopecia. However, what role does RCD play in HFs? Which cell types are prone to cell death [143]? Which genes can be targeted to treat this disorder? To obtain answers to these questions, further research is needed, and the role of RCD in HFSCs has garnered attention for the pathological and physiological processes in hair [144, 145]. It has been reported that the degree of HFSC damage determines whether alopecia is reversible [143]. The targets involved in RCD for improving HFSCs or improving HFSC-based therapy may provide novel strategies for skin-related diseases such as alopecia, skin cancer, skin inflammation, and skin wound healing.

#### Apoptotic pathways

To date, an emerging body of evidence has highlighted an important role for apoptosis of HFSCs [142, 146, 147]. For example, DNA damage caused by ionizing radiation causes premature senescence of HFs, which is associated with apoptosis of cells outside and inside the HFSC population [12]. A brief relevant review on the role of RCD in HFSCs is presented.

Apoptosis is a key RCD in which reversible cell damage is blocked by small-molecule inhibitors and a regulated process of cell death is initiated by multiple stresses, including DNA damage caused by radiation, reactive oxygen species (ROS), viral infection, and so on [148]. According to the inducing signals, the apoptotic pathway has been categorized into two forms: the intrinsic pathway initiated by intracellular stresses (*e.g.*, ROS and DNA damage) and the extrinsic pathway triggered by extracellular cues [149, 150]. There are various molecules involved in apoptosis (cytochrome C (cyt C), p53, caspases and Bcl-2). Among these molecules, caspases and Bcl-2 family proteins are the two key members that have also been thoroughly studied in HFSCs (shown in Fig. 7).

**Fig. 7:** The apoptotic pathway in HFSCs. There are two apoptotic pathways, namely, the intrinsic pathway initiated by intracellular stresses (*e.g.*, ROS and DNA damage) and the extrinsic pathway triggered by extracellular cues. **a** Intrinsic stressors upregulate the expression/activation of proapoptotic BCL-2 family members and suppress anti-apoptotic BCL-2 family proteins, resulting in MOMP. Intrinsic stressors can also induce the overexpression of proapoptotic proteins (*e.g*., NOXA (proapoptotic BH3-only protein, also known as PMAIP1 [phorbol-12-myristate-13-acetate-induced protein 1]), p53 upregulated modulator of apoptosis (PUMA), and apoptosis regulator Bcl-2-associated X protein (Bax)) in the p53-based apoptotic pathway, which is induced by the activation and stabilization of p53 through phosphorylation leading to its nuclear translocation, DNA binding and transcriptional initiation. Once MOMP is induced, cyt-c is released from the mitochondrial intermembrane and associates with caspase-9 and Apaf-1 to form apoptosomes, which can activate caspase-3 or caspase-7, causing apoptosis. **b** The extrinsic apoptotic pathway is triggered by the combination of the tumour necrosis factor receptor (TNFR) family members and specific TNF family ligands, leading to a caspase response. Once bound, TNFR/TNF undergoes a conformational change resulting in the recruitment of Fas-associated death domain (FADD) and subsequently pro-caspases-8 to form the death-inducing signalling complex (DISC). Finally, activated and cleaved caspase-3 leads to the occurrence of apoptosis, with characteristic changes such as phosphatidylserine plasma membrane exposure, DNA fragmentation, and the formation of apoptotic bodies. Remarkably, the intrinsic and extrinsic pathways are connected via the Bid protein. The T-shaped lines indicate inhibitory interactions involved in this pathway, and the solid arrows indicate activating interactions

### The intrinsic pathway of apoptosis

The intrinsic apoptotic pathway is defined by mitochondrial outer membrane permeabilization (MOMP). Intrinsic stressors upregulate the expression/activation of proapoptotic B cell lymphoma 2 (BCL-2) proteins and suppress anti-apoptotic BCL-2 family proteins, resulting in MOMP [151]. This outcome suggests that the BCL-2 family is a core element in intrinsic apoptosis [152, 153], in which pro-apoptotic BCL-2 proteins (*e.g.*, Bax and Bak) create pores in the outer mitochondrial membrane (OMM) to induce MOMP during apoptosis, while anti-apoptotic BCL-2 proteins inhibit this cascade (*e.g.,* Bcl-2, Bcl-x L, and Mcl-1) [154, 155]. Notably, intrinsic stressors can induce the overexpression of pro-apoptotic proteins (*e.g.,* NOXA (the pro-apoptotic BH3-only protein, also known as PMAIP1 [phorbol-12-myristate-13-acetate-induced protein 1]), p53 upregulated modulator of apoptosis (PUMA), and apoptosis regulator Bcl-2-associated X protein (Bax)) in the p53-based apoptotic pathway, which refers to the activation and stabilization of p53 by phosphorylation leading to its nuclear translocation, DNA binding and transcriptional initiation [156–159].

This delicate balance of BCL-2 family members contributes to the life of HFSCs. Upon induction of minor damage, HFSCs usually undergo anti-apoptotic progression, while irreversible damage may lead to cell elimination through apoptosis [160]. To ensure bulge homeostasis, HFSCs are continuously renewed, with new cells replacing differentiated or/and damaged cells, which are lost after wounding or chemotherapy-induced damage [159]. During extended periods of self-renewal and repair, HFSCs are at high risk for accumulating deleterious mutations. Therefore, they exhibit a powerful ability to resist damage, as indicated by high expression of *Bcl-2* (an anti-apoptotic gene) and transient stabilization of p53 [160]. A study has shown that IRS, matrix, and ORS keratinocytes undergo apoptosis in the catagen phase, whereas bulge HFSCs escape apoptosis [1, 25].

However, an increasing body of evidence indicates that permanent loss of hair regeneration can sometimes occur following the use of busulfan (Bu), etoposide, carboplatin, cyclophosphamide, docetaxel, paclitaxel or other drugs [161, 162]. These permanent hair loss conditions may be caused by a persistent change in DNA double-strand breaks in HFSCs, mostly in the DNA-replicating S phase [159]. Strategies to ensure that the damage is restricted to a range that can tolerated and to induce action, such as by triggering the upregulation of BCL-2 family genes to prevent permanent or irreversible damage under different conditions (*e.g.,* population, age, sex), remain to be further researched. Additionally, an in-depth study may reveal a clearer mechanism of apoptosis of HFSCs, which may include an unconventional signalling pathway in HFSCs, similar to other SCs.

Once MOMP is induced, cyt-c is released from the mitochondrial intermembrane and associates with caspase-9 and Apaf-1 to form apoptosomes, which can activate caspase-3 or caspase-7, causing apoptosis [163]. Remarkably, caspases are other pivotal components involved in apoptosis and can be functionally subdivided into two types: initiator caspases (caspase-8/9/10) and effector caspases (caspase-3/6/7) [164–166]. The initiator caspases interact through their large N-terminal pro-domain with a specific adaptor protein, leading to dimerization-induced activation for the cleavage of effector caspases. In contrast, effector caspases can spontaneously dimerize without need for cleaving a pro-domain [167, 168]. Among these caspases, caspase-3 is usually utilized as a biomarker for the detection of apoptosis [169]. In HFSCs, higher expression of caspase 3 has been found after irradiation-induced DNA damage [12]. Most important, caspases and Bcl-2 may be targets that regulate the apoptosis for HFSCs. For example, the Jian group revealed that a miR-149-5p inhibitor can suppress the proliferation and trigger the apoptosis of HFSCs, while miR-149-5p can upregulate the expression of Bcl-2 and downregulate caspase 3, as well as induce anti-apoptotic responses during superior-quality brush hair formation [170].

### The extrinsic pathway of apoptosis

The extrinsic apoptotic pathway is triggered by the combination of the tumour necrosis factor receptor (TNFR) family members and specific TNF family ligands, leading to a caspase response. Once induced, TNFR/TNF causes undergoes a conformational change resulting in the recruitment of Fas-associated death domain (FADD) and subsequently pro-caspases-8 to form the death-inducing signalling complex (DISC). Finally, activated and cleaved caspase-3 leads to apoptosis, with characteristic changes such as phosphatidylserine exposure to the outer plasma membrane, DNA fragmentation, and the formation of apoptotic bodies [171]. During wound healing, SCs near the wound seem to be awakened and activated to induce proliferation and differentiation needed for tissue repair. The conditional ablation of epidermal caspase-8 was identified as a cutaneous wound-healing response [172]. Additionally, a series of highly activated HFSCs have been found in *Casp8*-cKO skin, which suggests a strong association of caspase-8 and HFSCs [173]. Unfortunately, there are many obstacles to in-depth investigation, such as the truncated lifespan of the *Casp8*-cKO mouse (~ 20 days).

#### Other RCD mechanisms

Moreover, various types of RCD mechanisms have recently been identified along with conventional RCD mechanisms, such as apoptosis [174]. Moreover, RCDs can play an important role in skin. Among those mechanisms, autophagy, pyroptosis, ferroptosis, and necroptosis have tremendous significance in skin, which may suggest remarkable modulatory impacts on skin-related disease treatment. For example, autophagy, a starvation-induced cellular recycling pathway, is now regarded as a critical event in regulating the skin microenvironment [175]. Phosphatase and tensin homologue (PTEN), an upregulated target of BMP2, is involved in autophagy and can be translocated to the nucleus during oxidative stress, leading to autophagy [176, 177]. In HFSCs, autophagy can promote the differentiation of HFSCs through the BMP2/PTEN axis (a survival pathway, as explained above) [126]. This outcome suggests that the RCD can establish a certain relationship with survival signalling during the life of HFSCs, and cell death may not function as an adverse factor in HFSCs. Pyroptosis, a specific caspase-1-mediated inflammatory form of RCD [178, 179], is closely related to alopecia, and skin defects disrupt autoinhibition [180, 181]. Similarly, necroptosis is known as a RIPK1/RIPK3-mediated response [182–188], and the Juan group reported that targeting RIPK1 can prevent skin inflammation damage [189, 190]. Ferroptosis, an iron-dependent signalling pathway with characteristic iron accumulation and lipid peroxidation [191–193], was recently identified as a novel mechanism through a valuable new strategy to efficiently kill human skin melanoma cells [194]. However, there are few studies on the role of these kinds of RCD in HFSCs, which may be a potential approach to improve the microenvironment as well as their function during the life of HFSCs.

Notably, a complex network develops between various survival and death pathways contributing to the development of HFSCs. For example, Notch blockade can promote the proliferation and inhibit the differentiation of hHFSCs, while a significantly lower apoptosis rate has been found [97]. Additionally, it has been reported that, at the end of the telogen phase, HFSC apoptosis is closely associated with the secretion of the Wnt proteins that activate SC, thereby initiating the anagen phase [195]. In the present study, it was discovered that ocu-miR-205 promoted apoptosis and altered the expression of genes and proteins involved in the Wnt, Notch and BMP signalling pathways to promote the transition of HF from the growth phase to the regression and resting phases [196]. Under certain circumstances, cell death may not function as an adverse factor in HFSCs, and autophagy can promote the differentiation of HFSCs through the BMP2/PTEN axis (a survival pathway mentioned above) [126]. Gradually, studies have directed attention to the vital tole of RCD pathways involved in the development of HFSCs and their connection with survival signalling pathways, which is emerging as a practical and integrated network with signalling co-functions that maintain the niche. However, to discover the mechanisms by which the survival and death pathways are connected and the key molecules involved requires further study, not only to perfect the understanding of the network but also to enhance the applications of therapeutic targets.

## Clinical applications based on the survival and death pathways in HFSCs

With the development of SC engineering, it is critical to know how detailed survival and death signalling is involved in HFSCs during the HF cycle, which will contribute to better clinical guidelines, such as those directed towards improved strategies against cell death for better HFSC-based therapy. From a pragmatic perspective, these signalling pathways provide precise targets for practical use in manipulating HFSCs and even other SCs, enabling repair of pathological tissue or inhibition of abnormal proliferation (shown in Table 2).

**Table 2:** Clinical application via targeting the molecules involved in the survival or death signalling of HFSCs

Diseases	Strategies	Signalling pathway	Targeting molecules	Regulation (up/down)	Effects	Refs
Androgenic alopecia	Finasteride, oral	Wnt/β-catenin pathway	β-catenin GSK3-β	Up Down	Inhibiting 5-α-R, which inhibits the conversion of testosterone to DHT which is an inhibitor of Wnt signaling, to upregulate HFSCs proliferation and differentiation leading to hair follicle regeneration	[197, 198]
	Flutamide, topical	Wnt/β-catenin pathway	β-catenin	Up	Inhibiting androgen receptor which working with β-catenin can inhibit Wnt signaling, to upregulate HFSCs proliferation and differentiation leading to hair follicle regeneration	[199]
	Bicalutamide	Wnt/β-catenin pathway	β-catenin	Up	Inhibiting androgen, whose receptor working with β-catenin can inhibit Wnt signaling to upregulate HFSCs proliferation and differentiation leading to hair follicle	[199, 200]
	Fluridil, oral	Wnt/β-catenin pathway	β-catenin	Up	Inhibiting androgen receptor which working with β-catenin can inhibit Wnt signaling, stimulating HFSCs proliferation and differentiation to promote anagen	[199, 201]
	Cyproterone acetate, oral	Wnt/β-catenin pathway	β-catenin	Up	Inhibiting androgen receptor which working with β-catenin can inhibit Wnt signaling, to stimulate HFSCs proliferation and differentiation	[199, 202]
	Spironolactone, oral	Wnt/β-catenin pathway	β-catenin	Up	Reducing adrenal androgen, whose receptor working with β-catenin can inhibit Wnt signaling and competitively blocking androgen receptors, stimulating HFSCs proliferation and differentiation to arrest hair loss progression and achieve partial hair regrowth	[199, 203]
	Melatonin, topical	Wnt/β-catenin pathway	Wnt	Up	Inhibiting Wnt deacylase Notum, which can inactivate Wnt, to stimulate HFSCs proliferation and differentiation leading to increase of anagen hair	[204, 205]
	Dutasteride	Wnt/β-catenin pathway	β-catenin GSK-3β	Up Down	Inhibiting 5-α-R, which inhibits the conversion of testosterone to DHT which is an inhibitor of Wnt signaling, to upregulate HFSCs differentiation	[206]
	1α,25-dihydroxyvitamin D3, topical	Wnt/β-catenin pathway	Wnt-10b	Up	Stimulating HFSCs proliferation and differentiation, leading to outgrowth of hair shafts and higher maturation of regenerated follicles	[207]
	Tretinoin	Wnt/β-catenin pathway	β-catenin	Up	Stimulating HFSCs proliferation and differentiation, leading to hair regrowth	[208, 209]
	Platelet rich plasma, injective	Wnt/β-catenin pathway	β-catenin	Up	Stimulating HFSCs proliferation and differentiation to induce faster telogen-to-anagen transition	[210]
		Intrinsic apoptotic pathway	Bcl-2	Up	Upregulating Bcl-2 to inhibit apoptosis of HFSCs	[210]
	Baicalin	Wnt/β-catenin pathway	Wnt-3a, Wnt-5a, frizzled 7, disheveled 2, β-catenin	Up	Stimulating HFSCs proliferation and differentiation, increasing hair follicle development, to prevent androgenetic alopecia	[211, 212]
	Photobiomodulation or low-level laser (light) therapy (LLLT)	Wnt/β-catenin pathway	Wnt	Up	Stimulating HFSCs proliferation and differentiation to improve hair density and growth rate	[213]
			β-catenin	Up	Promoting hair regeneration through synergetic activation of β-catenin in HFSCs by ROS and paracrining Wnt by SKPs	[214]
	Transcutaneous implantation of valproic acid-encapsulated dissolving microneedles	Wnt/β-catenin pathway	β-catenin	Up	Stimulating HFSCs proliferation and differentiation to stimulate hair follicle regrowth	[215]
	Red Ginseng Oil	Wnt/β-catenin pathway	β-catenin, LEF-1	Up	Stimulating HFSCs proliferation and differentiation, inducing hair regrowth	[216]
		Shh pathway	Shh, Smoothened, Gli-1, Cyclin D1, and Cyclin E	Up	Stimulating HFSCs proliferation and differentiation, inducing hair regrowth	[216]
		Intrinsic apoptotic pathway	Bcl-2	Up	Inhibiting apoptosis of HFSCs, inducing hair regrowth	[216]
Chemotherapy-induced alopecia	Photobiomodulation or LLLT	Wnt/β-catenin pathway	Wnt	Up	Stimulating HFSCs proliferation and differentiation to improve hair density and growth rate	[213, 217]
	Immuvert/N-acetyl cysteine, topical	Apoptotic pathway	ROS	Down	Decreasing ROS production to reduce apoptosis to prevent cyclophosphamide/cytarabine-induced alopecia	[218]
	Calcitriol, 1,25-dihydroxyvitamin D-3 (Topitriol), topical	Wnt/β-catenin pathway	Wnt-10b	Up	Stimulating HFSCs proliferation and differentiation, leading to outgrowth of hair shafts and higher maturation of regenerated follicles	[207, 219]
Telogen effluvium	12-o-tetradecanoylphorbol-13-acetate (TPA)	Wnt/β-catenin pathway	Wnt-10b	Up	Stimulating HFSCs proliferation and differentiation to accelerate reentry of hair follicles into anagen phase	[6]
Inflammatory alopecias	N (1)-methylspermidine	Apoptotic pathway	ROS	Down	Reducing apoptosis of HFSCs; stimulating expression of the HFSC-associated keratin leading both anti-inflammatory and anti-oxidant effects, prolonging anagen	[220]
Alopecia	Tocotrienol	Wnt/β-catenin pathway	β-catenin	Up	Upregulating β-catenin by fourfold to stimulate HFSCs proliferation and differentiation, leading to hair follicular regeneration	[221, 222]
	3,4,5-tri-O-caffeoylquinic acid (TCQA)	Wnt/β-catenin pathway	Wnt, β-catenin	Up	Stimulating HFSCs proliferation and differentiation, promoting the initiation of the anagen phase of the hair cycle	[223]
	Loliolide	Wnt/β-catenin pathway	β-catenin	Up	Stimulating HFSCs proliferation and differentiation, inducing hair growth	[224]
	Sinapic acid	Wnt/β-catenin pathway	β-catenin	Up	Stimulating HFSCs proliferation and differentiation, inducing hair growth	[225]
	Costunolide	Shh pathway	Gli-1	Up	Stimulating HFSCs proliferation and differentiation, inducing hair growth	[226]
		Wnt/β-catenin pathway	β-catenin	Up	Stimulating HFSCs proliferation and differentiation, inducing hair growth	[226]
		BMP pathway	BMP1, BMP2, BMP6	Down	Stimulating HFSCs proliferation and differentiation, inducing hair growth	[226]
	Silibinin	Wnt/β-catenin pathway	Wnt-5a, LEF1	Up	Stimulating HFSCs proliferation and differentiation, promoting hair proliferation	[227]
	Ginkgolide B (GKB) and bilobalide (BB)	Wnt/β-catenin pathway	β-catenin	Up	Stimulating HFSCs proliferation and differentiation, promoting the cycle of hair follicles	[228]
	Morroniside, injective	Wnt/β-catenin pathway	Wnt-10b, β-catenin, LEF1	Up	Stimulating HFSCs proliferation and differentiation, accelerating the onset of anagen and delaying catagen	[229]
	Polygonum multiflorum extract, topical	Wnt/β-catenin pathway	β-catenin	Up	Stimulating HFSCs proliferation and differentiation, inducing anagen phase in resting hair follicles to promote hair growth	[230]
		Shh pathway	Shh	Up	Stimulating HFSCs proliferation and differentiation, inducing anagen phase in resting hair follicles to promote hair growth	[230]
	Nut oil from Prunus mira Koehne	Wnt/β-catenin pathway	Wnt-10b, β-catenin	Up	Stimulating HFSCs proliferation and differentiation, accelerating hair follicles	[231]
	Hot water extract of Thuja orientalis	Wnt/β-catenin pathway	β-catenin	Up	Stimulating HFSCs proliferation and differentiation, inducing an earlier anagen phase and prolonging the mature anagen phase	[232]
		Shh pathway	Shh	Up	Stimulating HFSCs proliferation and differentiation, inducing an earlier anagen phase and prolonging the mature anagen phase	[232]
	Human dermal stem/progenitor cell-derived conditioned medium	Wnt/β-catenin pathway	Wnt-3a, β-catenin	Up	Stimulating HFSCs proliferation to promote hair regeneration	[233]
Inflammation during burn injuries	Sirt1, gene upregulation	Apoptotic pathway	ROS	Down	Reducing apoptosis of HFSCs to enhance the survival of HFSCs in the inflammatory microenvironment	[234]
Inflammatory scalp diseases	N (1)-methylspermidine	Apoptotic pathway	ROS	Down	Reducing apoptosis of HFSCs; stimulating expression of the HFSC-associated keratin leading both anti-inflammatory and anti-oxidant effects	[220]
Psoriasiform-like skin inflammation	Imiquimod (IMQ), topical	Wnt/β-catenin pathway	Wnt	Up	Stimulating HFSCs activation	[235]
		BMP pathway	BMP4	Down	Stimulating HFSCs activation	[235]
Skin wound	Gut-derived human alpha defensin 5	Wnt/β-catenin pathway	Wnt1	Up	Increasing LGR + stem cell migration into wound beds, leading to enhanced healing, bacterial reduction, and hair production through the augmentation of key Wnt	[236]
Basal cell carcinoma	Vismodegib and function-blocking anti-LRP6 antibody	Shh pathway	Smoothened	Down	Leading to stop of the cancer growth	[237]
		Wnt/β-catenin pathway	LRP6	Down	Reducing the cell identity switch to avoid relapsing after treatment	[237]

### Alopecia

In medical practice, alopecia seems to be an exceedingly prevalent complaint, and the treatment is still difficult and frustrating due to the limited efficacy, long treatment length, and possible adverse side effects. HFSCs play important roles in appropriate hair recovery and regeneration, as indicated in cases of permanent hair loss, such as scarring alopecia, resulting from the irreversible loss of HFSCs [198]. Some alopecia, such as androgenic alopecia (AGA), is reversible because HFSCs are preserved [67]. Therefore, it seems necessary to improve the survival of HFSCs. Based on multiple causes of alopecia including the HFSC damage, a variety of strategies have been utilized for treating against alopecia, including SC-based therapy and biotechnology, platelet-rich plasma (PRP), drug treatment, and also placental extract, peptides, hormones, growth factors and cytokines, androgens and their analogs, stress-serum and chemotherapeutic agents, lipid-nanocarrier, light, electrical and electromagnetic field stimulation, and so on.

SC-based therapy and hair bio-engineering have risen tremendous expectations for alopecia treatment, which provides a new resource and advances hair growth. Clinically, the use of micrografts containing autologous human hair follicle mesenchymal stem cells (HF-MSCs) is considered as a safe and viable treatment alternative against alopecia [238, 239]. It has been reported that the injection of HFSCs preparations in AGA patients could increase their hair count and hair density up to baseline values [240].

Proponents of PRP approach suggest the benefits for improving the hair growth and increasing in hard/soft-tissue wound healing [241, 242]. PRP technology is based on the growth factors released from platelets, which could regulate multiple types of stem cells in the bulge of the HFs to induce the generation and development of new follicles [243]. The increased hair counts and total hair density, and increased epidermis thickness and of the number of HFs have been discovered after treating with PRP, almost in AGA patients [241, 244–246].

As for drug treatment, there are only two drugs, namely Minoxidil® and Finasteride®, which have been approved for the treatment of hair loss by the US Food and Drug Administration (FDA) [247]. Compared with Minoxidil® and Finasteride®, PRP presents as positive effects on AGA patients which is in absence of major side effects. So, PRP be may regarded as a safer and more effective alternative procedure to treat against alopecia [248].

The reversing the pathological mechanisms in various agents (both in PRP and SC-based therapy) are complex, which contribute to regeneration of HFs, or creating hair, or downregulation of hair loss [249]. For example, the activation of Wnt signalling in dermal papilla cells used in stimulating hair growth; MSC-derived signalling and growth factors obtained by platelets could utilized in the improvement of hair growth via regulating cellular proliferation through inducing cell growth (binding growth factors, such as PDGF, TGF-β, and VEGF), and HF development (Wnt activation), and suppress apoptotsis (Bcl-2 activation and release) [67, 249].

In the epidermis, overexpression of Wnt ligand can increase the number of regenerated HFs after wounding-induced folliculogenesis, providing a window for HF neogenesis in wounded tissue, hair loss and other degenerative skin disorders through Wnt protein signalling [250, 251]. Qiu et al*.* reported that TPA (12-o-tetradecanoylphorbol-13-acetate, a tumour promoter) can accelerate the re-entry of HFSCs into the anagen phase through various processes, such as the induction of Akt signalling to inhibit hair regeneration-related inhibitory signalling (*e.g*., FGF18) and then induction of Wnt/β-catenin to promote hair regeneration [6].

To prevent cell loss in HF induced by chemotherapy, two broad strategies are recommended: 1) preventing toxic drugs from reaching HFs and 2) protecting cells against death by inhibiting ROS, resisting cytotoxicity mediators and upregulating Bcl-2 expression to block apoptotic signalling [3]. Additionally, various drug candidates have largely been shown effective in improving alopecia treatments whose mechanism may relate to HFSCs; however, further research is needed, including investigations into ATP-sensitive potassium channel openers, 5-a-R inhibitors, androgen receptor antagonists, topical growth factors, a diverse selection of antioxidants and botanical extracts [3].

### Skin cancer

During the development of in-depth studies between molecular pathways and cancer, precise targeted therapy has been established to target key molecules that kill tumour cells and/or inhibit tumour progression. It has been reported that multiple HFSC populations readily develop BCC-like tumours in Ptch1-deleted mice, and targeting Shh signalling pathway components, such as using smoothened inhibitors (*e.g.*, vismodegib (Erivedge®) and sonidegib (Odomzo®), can treat BCC [88, 252]. Gαs-PKA has been found to play an important tumour suppressive role that limits the proliferation of HFSCs and maintains proper HF homeostasis with increased Shh signalling [253]. Cisplatin and mitomycin C DNA cross-linking agents have been utilized for the treatment of epithelial cancers to promote the apoptosis of rapidly cycling tumour cells as well as HFSCs, but some studies have discovered that chemotherapeutic DNA cross-linking agents can promote stem cell hyperplasia [254, 255]. Moreover, using DAPT (24-diamino-5-phenylthiazole, a Notch signalling blocker and γ-secretase inhibitor) can lead to promotion of HFSC proliferation and inhibition of differentiation through regulation of p21 and Wnt-10b [97]. γ-Secretase inhibitors have been contemplated for use as potential therapies for Notch-induced cancers. Although the multiple and complex mechanisms of resistance and side effects may challenge treatment, further understanding and continued research will provide an improved systemic treatment strategy.

### Skin inflammation

SC-based therapy is a promising tool for the treatment of burn injuries, whose treatment efficacy is seriously influenced by the inflammatory microenvironment in the damaged skin. To address this challenge, Sirtuin-1 (Sirt1) has been found to be an effective target to enhance the survival of HFSCs in the inflammatory microenvironment by inhibiting mitochondrial ROS overproduction, mitochondrial cyt-c liberation, and the upregulation of pro-apoptotic proteins [256]. The Yuval group showed that 0.5 µM N1-MeSpd had a strong effect on human HF cycling by prolonging the anagen phase, decreasing the apoptosis rate and stimulating the expression of HFSC-associated keratin, leading to both anti-inflammatory and anti-oxidant effects [220]. Other inflammatory-related disorders, such as psoriasis and atopic dermatitis, are also treated through these signalling pathways. For example, topical imiquimod (IMQ) application can induce psoriasiform-like skin inflammation via the reduced expression of the anagen-inhibiting factor BMP-4 and the upregulation of Wnt factors, leading to HFSC activation [235]. Multiple skin diseases are closely related to inflammation, which suggests targets for treating inflammation, such as reducing ROS levels, inhibiting the release of cyt C and regulating survival pathways.

### Skin wound healing

For scar-forming and regenerative skin wound healing, Shh signalling may be a potential target that plays a major role in preventing wounded fibroblasts from scarring by promoting and stimulating HFSC generation [121]. For skin wound healing, bioengineering revolved around the development of new autologous-technologies has led to considerable improvements, whereas skin appendages lost during injury are not regenerated [257–259]. Autologous non-activated platelet-rich plasma (A-PRP) or activated platelet-rich plasma (AA-PRP) have been utilized in wound healing. through autologous platelets derived growth factors aiming to aid the wound healing process. These factors could support in hair activation, induce cell differentiation, proliferation and neo-angiogenesis [259, 260].

Recently, a combination of culture-expanded HFSCs and skin-derived precursors (SKPs) was sufficient to regenerate de novo HFs through upregulation of BMP4 [261]. Moreover, an immune-related pathway known as the macrophage-TNF-induced AKT/β-catenin signalling pathway plays a crucial role in HFSCs to promote HF cycling and neogenesis after wounding, which provides a novel immune point [262]. Additionally, Wnt proteins may provide a mechanism for manipulating HF neogenesis after skin wounding. Wounding-induced folliculogenesis is abrogated after Wnt signalling is inhibited, whereas the number of regenerated HFs is upregulated through overexpression of the Wnt ligand [250]. Nonetheless, early intervention treatment in the developmental plasticity of HFSCs is necessary because SC status affecting tissue damage can be flexibly regained via early Wnt3a treatment ex vivo [263]. These targets seem to offer a good strategy for promoting skin wound healing, but the true curative effect is unsatisfactory, and the regeneration of skin through bioengineering is still a challenge that needs further study. Alternatively, co-network signalling may be a better approach, as might be achieved through the combined leverage of the Wnt and Shh signalling pathways.

## Conclusions

The balance between the survival and death of HFSCs contributes to the maintenance of a pool of HFSCs and the control of their abnormal proliferation, which is vital for tissue homeostasis and injury repair. Recent breakthroughs in novel single-cell profiling and spatial transcriptomics have led to more insights and greater understanding of the cell biology, structural and metabolic biochemistry and biological function of HFSCs from the gross and light microscopic levels to the molecular level. At the molecular level, complex and systematic signalling pathways in HFSCs have been presented for a better understanding of physiological and pathological (particularly for survival and death) processes, such as the Wnt, Shh, Notch, BMP, TGF, apoptotic, and autophagy pathways.

Notably, different signals lead to diverse characteristics during the life of HFSCs, Wnt/β-catenin can fuel HFSC activity for HF renewal, Shh signalling can improve quiescent-HFSCs proliferation, Notch signals can stop the differentiation programmes of HFSCs, BMP signals can modulate or reinforce the quiescence of HFSCs, the apoptotic pathway can respond to damage and induce self-cleaning. However, an abnormal intensity of signalling activation may lead to a suboptimal health status, such as in Wnt-induced cancer. Practically, the signalling pathways described provide effective therapeutic targets, and various drugs have been utilized for the treatment and/or the improvement of HFSC-based therapy.

Although much has been achieved through the targeting of key molecules for therapy, such as Shh inhibitors used to treat against BCC, there are still many challenges, such as determining the mechanistic framework in HFSCs, overcoming the limited efficacy of targeted drugs, shortening the length of treatments, and minimizing possible adverse side effects. Remarkably, the multifaceted signalling network and cell–cell and multiple system interactions, as well as the complex but practical integrated network in the niche, in the life of HFSCs have captured our attention. Overall, deeper knowledge of this network is key to a better understanding of HFSCs and results-oriented therapeutic targeting.

## Data Availability

Data sharing not applicable to this article as no datasets were generated or analysed during the current study.

## Abbreviations

AA-PRP: Activated Platelet-rich plasma
AGA: Androgenic alopecia
A-PRP: Autologous non-activated Platelet-rich plasma
APM: Arrector pili muscle
xin2: Axis inhibition protein 2
Bax: Bcl-2-associated X protein
BB: Bilobalide
BCC: Basal cell carcinoma
BCL-2: B cell lymphoma 2
bHLH: Basic helix-loop-helix
BMP: Bone morphogenetic proteins
BMPR: Bone morphogenetic protein receptor
Bu: Busulfan
Cdh: Congenital diaphragmatic hernia
Co-A: Coactivators
Co-R: Corepressor
cyt C: Cytochrome C
DAPT: 24-Diamino-5-phenylthiazole
DHT: Dihydrotestosterone
DISC: Death-inducing signalling complex
DP: Dermal papilla
Dvl: Disheveled
EGFR: Epidermal growth factor receptor
FADD: Fas-associated death domain
Fgf: Fibroblast growth factor
Flg: Filaggrin; Fox: Forkhead box
Foxp1: Forkhead box protein 1
Gli: Glioma-associated oncogene homolog
GPCR: G protein-coupled receptor
GSK-3β: Glycogen synthase kinase-3β
HDACs: Histone deacetylases
Hes: Hairy enhancer of the split
Hey: Hairy/enhancer-of-split related with YRPW motif
HFs: Hair follicles
HFSCs: Hair follicle stem cells
HG: Hair germ
hHFSC: Human hair follicle stem cells
IGFBP: Insulin-like growth factor-binding protein
IGFR: Insulin-like growth factor
IMQ: Topical imiquimod
IRS: Inner root sheath
Jag1: Jagged 1
K15: Keratin 15
KC: Keratinocytes
Lef: Lymphoid enhancer-binding factor
Lgr: Leucine-rich repeat-containing G protein-coupled receptor
Lhx: LIM homeobox
LLLT: Low-level laser (light) therapy
Lrp5/6: Receptors lipoprotein receptor-related protein
MAM: Mastermind
miRNAs, miRs: MicroRNAs
MOMP: Mitochondrial outer membrane permeabilization
NICD: Notch intracellular domain
OMM: Outer mitochondrial membrane
ORS: Outer root sheath
PDGF: Platelet-derived growth factor
PHLDA1: Pleckstrin homology-like domain family A member 1
PMAIP1: Phorbol-12-myristate-13-acetate-induced protein 1
PRP: Platelet-rich plasma
PTCH: Patched
Ptch1: Patched-1
PTEN: Phosphatase and tensin homologue
PUMA: P53 upregulated modulator of apoptosis
SC: Stem cell
sFRP-1: Secreted frizzled-related protein-1
Shh: Sonic hedgehog
Sirt1: Sirtuin-1
SKPs: Skin-derived precursors
Smo: Smoothened
Sox: SRY-related high-mobility-group box
TACs: Transient amplifying cells
Tcf: T-cell factor
TCQA: 3,4,5-Tri-O-caffeoylquinic acid
TDAG51: T cell death-associated gene 51
TGF-α: Transforming growth factor-α
TGF-β: Transforming growth factor-beta
TGM: Transglutaminase
Tmeff1: Tomoregulin-1
TNFR: Tumour necrosis factor receptor
TPA: 12-O-tetradecanoylphorbol-13-acetate
UV: Ultraviolet
VEGF: Vascular endothelial growth factor
